# MicroRNA-377 Suppresses Cell Proliferation and Invasion by Inhibiting TIAM1 Expression in Hepatocellular Carcinoma

This article has been retracted.

**DOI:** 10.1371/journal.pone.0117714

**Published:** 2015-03-04

**Authors:** Guolin Chen, Lu Lu, Chang Liu, Lei Shan, Di Yuan

**Affiliations:** 1 The First Ward of Infection Department, the First Clinical Hospital Affiliated to Harbin Medical University, Harbin, Heilongjiang, China; 2 Department of Medical Oncology, The Fourth Affiliated Hospital of Harbin Medical University, Harbin, Heilongjiang, China; 3 Clinical Laboratory, The First Clinical Hospital Affiliated to Harbin Medical University, Harbin, Heilongjiang, China; H.Lee Moffitt Cancer Center & Research Institute, UNITED STATES

## Abstract

Increasing evidence has suggested that microRNAs (miRNAs) play an important role in the initiation and progression of hepatocellular carcinoma (HCC). Here, we identified a novel tumor suppressive miRNA, miR-377, and investigated its role in HCC. The expression of miR-377 in HCC tissues and cell lines was detected by real-time reverse-transcription PCR. The effects of miR-377 on HCC cell proliferation and invasion were also investigated. Western blot and luciferase reporter assay were used to identify the direct and functional target of miR-377. The expression of miR-377 was markedly downregulated in human HCC tissues and cell lines. MiR-377 can dramatically inhibit cell growth and invasion in HCC cells. Subsequent investigation revealed that T lymphoma invasion and metastasis 1 (TIAM1) was a direct and functional target of miR-377 in HCC cells. Overexpression of miR-377 impaired TIAM1-induced promotion of proliferation and invasion in HCC cells. Finally, miR-377 is inversely correlated with TIAM1 expression in human HCC tissues. These findings reveal that miR-377 functions as a tumor suppressor and inhibits the proliferation and invasion of HCC cells by targeting TIAM1, which may consequently serve as a therapeutic target for HCC patients.

## Introduction

Hepatocellular carcinoma (HCC) is one of the most aggressive and common malignancies, with high mortality and prevalence rates in East Asian countries including China[1]. Despite therapeutic advances, the 5-year survival rate of HCC patients is still only approximately 5%, with exceeding 600,000 people dying of HCC each year[2]. HCC is the result of a complex, multi-step process associated with genetic and epigenetic changes[3,4]. Hence, it is important to develop novel strategies for the early diagnosis, prediction of the prognosis, and the treatment of patients with HCC.

microRNAs (miRNAs) are a group of small noncoding RNAs averaging 20 to 24 nucleotides and mediate translational suppression or cleavage of their target mRNAs by binding to complementary sites in their 3′-UTR[5–7]. Since the initial observation, over 1000 miRNAs have been determined in mammals, but their detailed roles in cancers still need investigation[8,9]. Recently, increasing evidences have suggested that miRNAs participate in the regulation of diverse processes such as tumor initiation, promotion, and progression, and their deregulation or dysfunction plays critical roles in cancer development and clinical outcomes of cancer patients[10–14].

In the present study, we explored the potential roles of miR-377 in HCC development. The expression of miR-377 in clinically resected human HCC tissues was evaluated, and the correlation between miR-377 deregulation and HCC progression was analyzed. Furthermore, the roles of miR-377 in HCC development and the underlying mechanisms were investigated. Our data indicate the role of miR-377 in the control of cell growth and invasion in HCC, and suggest the potential therapeutic application of miR-377 for HCC patients.

## Materials and Methods

### Ethics Statement

All patients or patients’parents on behalf of the children agreed to participate in the study and gave written informed consent. This study and consent was approved by the ethical board of the institute of The first clinical hospital affiliated to Harbin Medical University and complied with Declaration of Helsinki.

### Hepatocellular carcinoma tissues

A total of 50 frozen primary tumor samples and corresponding non-tumorous tissue samples (located >3cm away from the tumor) were obtained from HCC patients were obtained from patients with hepatectomy undergoing surgery at The first clinical hospital affiliated to Harbin Medical University. The TNM classification of the Union for International Cancer Control (UICC) was used. None of the patients received radiotherapy or chemotherapy before surgery. The characteristics of patients are described in Table S1.

### Cell lines and Cell culture

The human HCC cell lines HepG2, SMMC7721 Hep3B and Bel7402 as well as normal human hepatocyte, HL-7702, were purchased from American Type Culture Collection (ATCC, Mannasas, VA, USA) and cultured in Dulbecco’s modified Eagle’s medium (DMEM, Gibco, USA) containing 10% foetal bovine serum (HyClone, USA) at 37°C in a humidified chamber supplemented with 5% CO2.

### Northern blot analysis

The analysis was performed according to a previous report with some modifications[15]. Total RNA (20 μg) was separated on 12.5% denaturing (7 mol/L urea) PAGE and then transferred onto Biodyne Nylon Transfer Membranes (0.2 mm; Pall Corp.) using a vacuum blotting system (GE Healthcare). The membrane was dried and UV cross-linked. The blots were prehybridized at 35°C for 30 minutes in hybridization buffer (GE Healthcare), and then each ^32^P-labeled LNA probe was added and incubated at 60°C for 2 hours. The membranes were washed twice in 2×SSC with 0.1% SDS at 60°C for 10 minutes.

### Quantitative Reverse Transcription-PCR

Total RNA containing miRNA and mRNA was extracted from cell lines or tissues using Trizol reagent (Invitrogen, Carlsbad, CA, USA), according to the manufacturer’s instructions. The expression of mature hsa-mir-377 and of U6 RNA, as housekeeping gene, was assayed using the TaqMan miRNA Assays (Applied Biosystems) as described previously. Real-time PCR was done in triplicate for each case using the standard TaqMan miRNA assays protocol on the ABI PRISM 7900 Sequence Detection System (Applied Biosystems). miRNA expression was measured using Ct (threshold cycle). The ΔΔCt method for relative quantitation of gene expression was used to determine miRNA expression levels. The ΔCt was calculated by subtracting the Ct of U6 RNA from the Ct of the miRNA of interest. Fold change was generated using the equation 2-ΔΔCt. The expression level of GAPDH was used as an internal control for mRNA expression.

### Oligonucleotide transfection

The miR-377 mimics, miR-377 inhibitor and their controls were synthesized by GenePharma (Shanghai, China) and transfected into the cells to a final oligonucleotide concentration of 20 nmol/L. All cell transfections were introduced by Lipofectamine 2000 (Invitrogen) according to the manufacturer’s instructions.

### Cell proliferation and invasion assays

For analysis of cell proliferation, cells were seeded into 24-well plates at 8×10^3^ cells/well. Cells were incubated in 10% Cell Counting Kit-8 (CCK-8; Dojindo, Kumamoto, Japan) and diluted in normal culture medium at 37°C until visual color conversion occurred. The proliferation rate was determined at 0, 24, 48, and 72 h after transfection. The absorbance in each well was measured with a microplate reader set at 450 nM. For analysis of cell invasion, the transwell chambers were coated with Matrigel (BD Biosciences, San Jose, CA, USA) and incubated at 37°C for 3 h, allowing it to solidify. After 24 h of transfection, 4×10^5^ cells suspended in serum-free DMEM were added to the upper chamber, and medium containing 10% FBS was added to the lower chamber. After 24 h, invasive cells located on the lower surface of the chamber were stained. Three independent experiments were performed.

### Luciferase assay

HepG2 cells were seeded in 24-well plates (1×105 cells/well) and incubated for 24 h before transfection. For the reporter gene assay, the cells were cotransfected with 0.5 μg of pGL3-TIAM1–3’UTR or pGL3- TIAM1–3’UTR Mut plasmid, 0.05 ng of the phRL-SV40 control vector (Promega, USA), and 100 nM miR-377 or control RNA using Lipofectamine 2000 (Invitrogen, USA). The firefly and renilla luciferase activities were measured consecutively through a dual luciferase assay (Promega, USA) 24 h after transfection.

### Western blot

Cells were harvested in ice-cold PBS 48 h after transfection and lysed on ice in cold-modified radioimmunoprecipitation buffer supplemented with protease inhibitors. Protein concentration was determined by the BCA Protein Assay Kit (Bio-Rad, Italy), and equal amounts of protein were analyzed by SDS-PAGE. Gels were electro blotted onto nitrocellulose membranes (Millipore, USA). Membranes were blocked for 2 h with 5% non-fat dry milk in Tris-buffered saline containing 0.1% Tween-20, and incubated at 4°C overnight with primary antibody. Detection was performed using peroxidase-conjugated secondary antibodies and the enhanced chemiluminescence system (ECL) (Millipore, USA). Primary antibodies used were TIAM1 (Cell Signaling Technology Inc., Danvers, MA, USA), and GAPDH (Zhong-Shan JinQiao, China).

### Statistical analysis

Each experiment was repeated at least three times. Statistical analyses were performed using SPSS 15.0. Data are presented as the mean ± standard deviation. Statistical analyses were performed with either an analysis of variance (ANOVA) or Student’s t-test, and the statistical significance level was set at α = 0.05 (two-side).

## Result

### miR-377 is downregulated in HCC cell lines

To explore the expression and significance of miR-377 in HCC carcinogenesis, we measured the expression of miR-377 in four human HCC cell lines (HepG2, SMMC7721 Hep3B and Bel7402) and HL-7702, a normal human hepatocyte. qRT–PCR showed that miR-377 expression was significantly decreased in HCC cell lines compared with HL-7702 (Fig. 1A). We further quantified the expression level of miR-377 in four human HCC cell lines (HepG2, SMMC7721 Hep3B and Bel7402) and HL-7702 using northern blot (Fig. 1B). The results also showed that the expression level of miR-377 was significantly decreased in HCC cell lines compared with HL-7702.

**Fig 1:** MiR-377 is downregulated in HCC cell lines. (A) Downregulation of miR-377 expression was in HCC cell lines. Relative expression of miR-377 in four HCC cell lines (HepG2, SMMC7721 Hep3B and Bel7402) and one normal human hepatocyte (HL-7702) was determined by qRT-PCR. U6 snRNA was used as internal control. (B) Northern blot analysis of miR-377 in four HCC cell lines (HepG2, SMMC7721 Hep3B and Bel7402) and one normal human hepatocyte (HL-7702). U6 snRNA was also detected as a loading control.

### Expression of miR-377 in clinical HCC patients and correlation analysis with clinicopathological characteristics

Among 50 cases of tumor tissues, 43 cases exhibited decreased miR-377 expression compared with the adjacent normal tissues (86%, 43 of 50, Fig. 2A). Further, statistical analysis demonstrated that the expression of miR-377 in HCC tissues was much lower relative to normal tissues (Fig. 2B). Low levels of miR-377 expression were associated with pTNM stage (Fig. 2C). Furthermore, tissues from lymph node metastases have lower levels of miR-377 compared with primary HCC tissues and the adjacent normal tissue, indicating an inverse relationship between the expression of miR-377 and the metastatic status of HCC tissues (Fig. 2D).

**Fig 2:** Expression of miR-377 in clinical HCC patients and correlation analysis with clinicopathological characteristics. (A) miR-377 was detected in 50 pairs of HCC tissues and its adjacent normal controls by quantitative RT-PCR. Data are presented as log2 of fold change of HCC tissues relative to adjacent normal regions. U6 snRNA was used as internal control. (B) Relative miR-377 expression levels in HCC tissues and adjacent normal tissues were determined by qRT-PCR. (C) The Statistical analysis of the association between miRNA level and pTNM stage (I, II, III and IV). (D) The relative expression of miR-377 in adjacent normal tissues, primary HCC tissues and lymph node metastatic tissues from 10 patients. *p<0.05, and **p<0.01, *** p<0.001.

### miR-377 inhibits HCC cell proliferation and invasion

First, qRT-PCR was performed to measure the level of miR-377 in HepG2 cells after transfection. We found that miR-377 expression was increased in transfected HepG2 cells using miR-377 mimics (Fig. 3A), and the miR-377 expression was decreased in transfected HepG2 cells using miR-377 inhibitor (Fig. 3B). The CCK-8 proliferation assay showed that the growth rate was reduced in HepG2 cells transfected with miR-377 mimics compared with cells transfected with scramble mimics or untreated (Fig. 3C). Meanwhile, the growth rate was increased in HepG2 cells transfected with miR-377 inhibitor compared with cells transfected with control mimics or untreated (Fig. 3D). The invasiveness of cells transfected with miR-377 mimics was dramatically decreased compared with the scramble group and control group cells and the invasiveness of cells transfected with miR-377 inhibitor was dramatically increased compared with the scramble group and control group cells (Fig. 3E).

**Fig 3:** MiR-377 inhibits HCC cell proliferation and invasion. (A) Real-time RT-PCR analysis of miR-377 in HepG2 cells upon transfection of miR-377. The expression of miR-377 in HepG2 cells transfected with miR-377 mimics was up-regulated. U6 snRNA was used as internal control. (B) The expression of miR-377 in HepG2 cells transfected with miR-377 inhibitor was down-regulated. U6 snRNA was used as internal control. (C) Invasion analysis of HepG2 cells after treatment with miR-377 mimics, inhibitors or scramble or control; the relative ratio of invasive cells per field is shown below, *p<0.05, ** p<0.01, and ***p<0.001.

### miR-377 downregulated TIAM1 through interaction with its 3’-untranslated region

As a potential miR-377 target, TIAM1 was selected for further assessment because PicTar predicted complementarity between miR-377 and the TIAM1 3’-UTR (Fig. 4A). To prove that miR-377 directly targets the TIAM1 3’UTR, we performed luciferase reporter gene assays. Ectopic of miR-377 remarkably reduced luciferase activity in the TIAM1 wild-type reporter gene but not the mutant TIAM1 3’UTR, indicating that miR-377 directly targeted the TIAM1 3’UTR (Fig. 4B). We also found that the mRNA level of TIAM1 was substantially decreased after transfection miR-377 mimics and the mRNA level of TIAM1 was increased after transfection miR-377 inhibitor using qRT-PCR (Fig. 4C). Consistent with this result, the ability of miR-377 to regulate the expression of the TIAM1 protein was verified by western blotting (Fig. 4D).

**Fig 4:** MiR-377 downregulates TIAM1 through interaction with its 3’-untranslated region. (A) Schematic representation of TIAM1 3’UTR was showing the putative miR-377 target site. (B) Relative luciferase activity of the indicated TIAM1 reporter construct in HepG2 cells is shown. Firefly luciferase values were normalized to Renilla luciferase activity and plotted as relative luciferase activity. (C) RT-PCR analysis was performed to examine the effects of miR-377 on TIAM1 expression in HepG2 cells. Ectopic expression of miR-377 significantly decreased HepG2 transcripts. GAPDH was used as internal control. (D) Western blotting was performed to examine the effects of miR-377 on the expression of TIAM1. GAPDH was also detected as a loading control.

Restoration of miR-377 inhibits TIAM1-mediated HCC cell proliferation and invasion Western blot of TIAM1 in the HepG2 cells transfected with the pcDNA-TIAM1 or vector control showed that pcDNA-TIAM1 could enhance the TIAM1 protein expression (Fig. 5A). The CCK-8 proliferation assay and invasion assay showed that overexpression of TIAM1 promote the HCC cell proliferation and invasion. When miR-377 and pcDNA-TIAM1 were cotransfected into HepG2 cells, miR-377 expression significantly reduced the TIAM1-induced HCC cell proliferation and invasion (Fig. 5B and C).

**Fig 5:** Restoration of miR-377 inhibits TIAM1-mediated HCC cell proliferation and invasion. (A) Western blotting was performed to examine the effects of pCDNA-TIAM1 on the expression of TIAM1. GAPDH was also detected as a loading control. (B) The cell growth in HepG2 co-transfected with either miR-377 mimic or scramble and 2.0 μg pCDNA- TIAM1 or pCDNA empty vector using CCK-8 proliferation assay. (C) The cell invasive in HepG2 co-transfected with either miR-377 mimic or scramble and 2.0 μg pCDNA- TIAM1 or pCDNA empty vector using invasion assay. *p<0.05, ** p<0.01, and ***p<0.001.

### miR-377 and TIAM1 are inversely expressed in HCC specimens

qRT–PCR has shown that TIAM1 expression was higher in HCC cell lines (HepG2, SMMC7721 Hep3B and Bel7402) compared with HL-7702 (Fig. 1A). The protein levels of TIAM1 were also higher in HCC cell lines compared with HL-7702 using western blot (Fig. 6B). Compared with the low expression of miR-377 in HCC tissues, the TIAM1 mRNA was expressed at higher levels (95%) (19/20) in tumor tissues compared with normal tissues (Fig. 6C). As shown in Fig. 6D, when the TIAM1 levels were plotted against miR-377 expression, a significant inverse correlation was obtained (two-tailed Pearson’s correlation analysis, r^2^ = -0.486; p<0.01).

**Fig 6:** MiR-377 and TIAM1 are inversely expressed in HCC specimens. (A) Relative expression of TIAM1 in four HCC cell lines (HepG2, SMMC7721 Hep3B and Bel7402) and one normal human hepatocyte (HL-7702) was determined by qRT-PCR. GAPDH was used as internal control. (B) Western blotting was performed to examine the TIAM1 protein expression in four HCC cell lines (HepG2, SMMC7721 Hep3B and Bel7402) and one normal human hepatocyte (HL-7702) was determined by qRT-PCR. GAPDH was used as loading control. (C) qRT-PCR analysis of TIAM1 expression in 20 pairs HCC tissues and their corresponding adjacent normal tissues. The expression of TIAM1 was normalized to GAPDH. (D) Analysis of correlation of miR-377 and TIAM1 expression in HCC tissues. (Two-tailed Pearson’s correlation analysis, r^2^ = -0.486; p<0.01). Data was presented as log 2 of fold change of HCC tissues relative to non-tumor adjacent tissues.

## Discussion

Recent studies have revealed that miRNAs act as an important regulator of gene expression at the post-transcriptional level and regulates a wide range of physiological and developmental processes[16–19]. Over the past several years, it has become clear that deregulated of miRNAs contribute to the development of most human cancers such as gastric cancer, bladder cancer and breast cancer, which they act as either oncogenes or tumor suppressors[20–23]. In the present study, we investigated the role of miR-377 in human HCC development. We found that the expression of miR-377 was decreased in all four HCC cell lines compared with HL-7702, a normal human hepatocyte. Furthermore, miR-377 was downregulated in advanced stages of HC, indicating its possible involvement in both oncogenic transformation and tumor metastasis. We subsequently confirmed that miR-377 significantly suppressed HCC cell proliferation and invasion. TIAM1 was identified as a critical downstream target of miR-377. We revealed that TIAM1 was upregulated in HCC cells, and exogenous miR-377 downregulated the expression of TIAM1 protein. Furthermore, luciferase reporter assays revealed that miR-377 could directly target the 3’-UTR of TIAM1 mRNA. Our findings suggest that miR-377 has a fundamental role in HCC tumorigenesis, such as cancer cell proliferation and invasion.

Previous studies have shown that miR-377 plays a critical role in the pathogenesis of diabetic nephropathy in both human cell lines and mouse models by regulating PAK1, SOD1, and SOD2 protein expression, leading to increased fibronectin production[24]. Another research demonstrated that miR-377 was involved in the regulation of HO-1 expression during hemolysis[25]. Moreover, miR-377 was also deregulated in some cancers, including late-stage and high-grade ovarian cancer, metastatic prostate cancer, breast cancer and splenic marginal zone lymphoma[26–29]. Recently, Zhang et al has shown that miR-377 inhibited proliferation and invasion of human glioblastoma cells by directly targeting specificity protein 1[30]. However, the role of miR-377 in HCC development and progression remains unclear. Our study showed that miR-377 was frequently downregulated in both HCC tissues and cell lines. Moreover, restoration of miR-377 can reduce HCC cell proliferation and invasion. These results suggest that miR-377 might act as a tumor suppressor gene whose down-regulation contributes to the progression and metastasis of HCC.

To explore the molecular mechanism by which miR-377 suppresses HCC cell line growth and invasion, we identified TIAM1 as a direct target of miR-377 in HCC cells. TIAM1, a member of the Dbl gene family of guanine nucleotide exchange factors (GEFs), was first identified by proviral tagging in combination with in vitro selection for invasiveness from murine leukemia cells[31]. TIAM1 has a major influence on various biological processes including cell migration and adhesion[32]. Alterations expression of Tiam1 may contribute to tumorigenesis and carcinoma progression in many types of human cancers[33]. Overexpression of TIAM1 is considered to be a new potential or even an independent predictor of poor prognosis for clinical patients[34]. Increasing evidences have shown that Tiam1 is a metastasis related gene of a variety of cancers, such as colorectal cancer, breast cancer, prostate cancer, lung cancer and renal cell carcinoma[35–41]. Moreover, previous studies proved the overexpression of Tiam1 in HCC tissues compared to the adjacent normal tissues[42]. Tiam1 showed a higher frequency of being overexpressed in HCC patients with metastasis than those without metastasis[43]. Moreover, survival analysis showed that the Tiam1 overexpression group had a significantly shorter overall survival time than the Tiam1 downexpression group. Multivariate analysis showed that Tiam1 expression was a significant and independent prognostic parameter for HCC patients[43,44]. However, the underlying mechanisms are unclear. In this study, we identified TIAM1 as a direct and functional target of miR-377. We confirmed the positive effects of TIAM1 protein on HCC cell proliferation and invasion in vitro. Moreover, miR-377-kmediated suppression of TIAM1 depended on the 3’-UTR. Finally, TIAM1-induced cell proliferation and invasion were reversed by miR-377. Taken together, these results establish a functional connection between miR-377 and TIAM1, and confirm that miR-7 functions as an anti-metastatic miRNA in HCC cells by targeting TIAM1. Moreover, we also found that miR-377 expression in HCC tissues correlated inversely with TIAM1 expression. The ability of miR-377 to target TIAM1 might be one mechanism underlying the post-transcriptional control of TIAM1.

In conclusion, our study indicates that miR-377 inhibits HCC cancer cells by negatively regulating the TIAM1 gene. Our findings also underscore the clinical potential of miR-377 in HCC treatment and support the development of effective therapeutic strategies that target miR-377 (or its targets such as TIAM1) by a genetic or pharmacological approach.
